# Survival Prediction Model for Patients with Esophageal Squamous Cell Carcinoma Based on the Parameter-Optimized Deep Belief Network Using the Improved Archimedes Optimization Algorithm

**DOI:** 10.1155/2022/1924906

**Published:** 2022-07-08

**Authors:** Yanfeng Wang, Wenhao Zhang, Junwei Sun, Lidong Wang, Xin Song, Xueke Zhao

**Affiliations:** ^1^School of Electrical and Information Engineering, Zhengzhou University of Light Industry, Zhengzhou 450000, China; ^2^State Key Laboratory of Esophageal Cancer Prevention & Treatment and Henan Key Laboratory for Esophageal Cancer Research of the First Affiliated Hospital, Zhengzhou University, Zhengzhou 450066, China

## Abstract

Esophageal squamous cell carcinoma (ESCC) is one of the highest incidence and mortality cancers in the world. An effective survival prediction model can improve the quality of patients' survival. Therefore, a parameter-optimized deep belief network based on the improved Archimedes optimization algorithm is proposed in this paper for the survival prediction of patients with ESCC. Firstly, a combination of features significantly associated with the survival of patients is found by the minimum redundancy and maximum relevancy (MRMR) algorithm. Secondly, a DBN network is introduced to make predictions for survival of patients. Aiming at the problem that the deep belief network model is affected by parameters in the construction process, this paper uses the Archimedes optimization algorithm to optimize the learning rate *α* and batch size *β* of DBN. In order to overcome the problem that AOA is prone to fall into local optimum and low search accuracy, an improved Archimedes optimization algorithm (IAOA) is proposed. On this basis, a survival prediction model for patients with ESCC is constructed. Finally, accuracy comparison tests are carried out on IAOA-DBN, AOA-DBN, SSA-DBN, PSO-DBN, BES-DBN, IAOA-SVM, and IAOA-BPNN models. The results show that the IAOA-DBN model can effectively predict the five-year survival rate of patients and provide a reference for the clinical judgment of patients with ESCC.

## 1. Introduction

Cancer is the second leading cause of death in the world and poses a great danger to human health [1, 2]. There will be approximately 19.29 million new cancer cases and 9.95 million cancer deaths worldwide in 2021 [3]. Esophageal cancer is the sixth most common cause of cancer-related death worldwide, including esophageal squamous cell carcinoma and esophageal adenocarcinoma [4]. More than 90% of esophageal cancers are esophageal squamous cell carcinoma (ESCC). The pathology of esophageal squamous cell carcinoma is complex, and it is often found at an advanced stage, which brings a huge burden to the patient's family [5, 6]. In recent years, the incidence of esophageal squamous cell carcinoma has been increasing [7], and the mortality rate is still high [8, 9].

One of the most fundamental difficulties in the treatment of ESCC is the lack of effective methods for predicting survival risk [10, 11]. Currently, with the more in-depth research on ESCC and the continuous development of medical technology [12], the use of various types of intelligent systems in esophageal cancer diagnosis is increasing [13]. The treatment methods and treatment concepts for patients with ESCC have continued to rise [14]. However, as with other malignancies, the incidence of patients with ESCC is increasing. Even for professional doctors, it is difficult to judge the patient's ultimate risk of survival [15].

Generally, blood indicators, age, and TNM stage information are considered related to the survival rate of cancer patients, and they are often used to predict the survival status of patients [16–18]. In recent years, with the continuous progress of machine learning technology, more and more intelligent algorithms are proposed and applied in multiple fields [19–21]. In the medical field, the research on the survival risk of cancer patients has become a popular research content [22]. A reasonable survival prediction model will effectively improve the survival of cancer patients. Essentially, the cancer patient survival prediction model is a classification problem [23], including the screening of datasets and analyzing the connections between the data. So far, many data mining methods have been proposed in the literature to predict the survival status of esophageal cancer patients [24, 25]. In [26], 90 breast cancer risk miRNAs are predicted based on the proposed DMTN by using the SVM classifier, which obtained an AUV of 0.9633. The method of backpropagation artificial neural network is adopted to predict whether postoperative fatigue occurred in patients undergoing gastrointestinal tumor surgery in [27], and the accuracy rate reached 0.872.

The above approach based on shallow architecture achieves good performance in cancer prediction problems. However, since the classification accuracy of shallow learning depends largely on the quality of the extracted features, it may cause problems when dealing with more complex applications [28]. In fact, for high latitude and complex cancer patient data, it is not sufficient to use simple traditional shallow architecture to solve it [29]. Correspondingly, the deep learning model has multiple nonlinear network structures, which enable it to extract the features of the original data from the hidden layer step by step and improve the classification and prediction accuracy of the model [30, 31]. Therefore, a network structure with deeper layers is preferred.

Deep learning is a new direction in the field of machine learning that models high-level abstractions in input data with hierarchies and multiple layers [32, 33]. Through the establishment of artificial neural network with a network hierarchy, multiple layers gradually extract higher-level features from the original input for learning. Different types of deep neural networks for classification prediction have been used in multiple literatures [34–36]. DBN is a probabilistic generative network, which is considered more suitable for prediction of cancer classification with high feature similarity and complexity [37]. However, in the process of building DBN, improper parameter setting will lead to the instability of the model and the problem of poor classification accuracy. Often, the selection of parameters still relies on the experience of experts to be manually tuned. Aiming at the above problems, a cancer patient survival prediction model based on the improved Archimedes optimization algorithm (IAOA) to optimize DBN parameters is proposed.

In this paper, seventeen blood indicators, age, and TNM staging information of 298 patients with ESCC are studied. Firstly, the clinical data of cancer patients are selected by the minimum redundancy and maximum relevancy algorithm, and the feature indexes are sorted according to their importance. A combination of eleven indicators is selected that is significantly associated with patient survival, which is verified by the Cox regression method in the SPSS software. Secondly, the IAOA is introduced to optimize the parameters in the DBN network training process to improve the stability and classification accuracy of the DBN model. Finally, a survival prediction model of patients with ESCC based on IAOA-DBN is established. The above eleven related indicators are used as inputs, and the five-year survival rate of the patient is used as output. The prediction accuracy rate of IAOA-DBN is better than the existing AOA-DBN, SSA-DBN, PSO-DBN, BES-DBN, IAOA-SVM, and IAOA-BPNN. Therefore, the method for survival diagnosis of patients with ESCC proposed in this paper can accurately predict the survival level of patients. The main contributions of this article can be summarized as follows:

1. A combination of eleven indicators is found based on minimum redundancy and maximum relevancy feature selection, which is verified to be significantly associated with survival in patients with ESCC
2. The proposed method uses IAOA to optimize the parameters of the DBN, which effectively improves the stability and classification accuracy of the DBN network. The problem that AOA tends to fall into local optimum and low convergence accuracy is effectively improved by the IAOA. Through the establishment of the IAOA-DBN model, the five-year survival rate of patients with ESCC is effectively predicted

This work is presented as follows. In Section 2, the original data is analyzed, and a combination of multiple indicators that is significantly related to patient survival is found based on minimum redundancy and maximum relevancy algorithm. An improved Archimedes algorithm is proposed in Section 3, which can effectively improve the optimization accuracy and stability of AOA. In Section 4, a survival prediction model based on IAOA-DBN is proposed, which can effectively predict the five-year survival rate of patients with ESCC. In Section 5, the conclusions of this article are presented.

## 2. Dataset Analysis

### 2.1. Data Introduction

The clinical data of 298 patients with ESCC used in this article are from patients who were treated in the First Affiliated Hospital of Zhengzhou University from January 2007 to December 2018. The clinical information includes seventeen blood indicators, age, and TNM staging information. The seventeen blood indicators are basophil count (BASO), eosinophil count (EO), fibrinogen (FIB), platelet count (PTL), albumin (ALB), hemoglobin concentration (HGB), white blood cell count (WBC), monocyte count (MONO), activated partial thromboplastin time (APTT), globulin (GLOB), red blood cell count (RBC), prothrombin time (PT), lymphocyte count (LYMPH), neutrophil count (NEUT), total protein (TP), international normalized ratio (INR), and thrombin time (TT). The population proportion information of the dataset is shown in Table 1. Information of seventeen blood indicators is shown in Table 2.

Among all patients, 147 patients survived more than five years, 151 patients survived less than five years, and the data are evenly distributed. The age distribution of the patients ranged from 38 to 82 years, including 190 male patients and 108 female patients. In addition, the selected patients should have complete treatment records and be followed up for more than six months.

### 2.2. Minimum Redundancy and Maximum Relevancy Algorithm

The minimum redundancy and maximum relevancy (MRMR) algorithm [38] is a typical feature selection method. The purpose of MRMR is to select the features with the minimal redundancy and the maximal relevance with the class label. The relevance between features and class labels is represented by mutual information. The mutual information is calculated as Equation (1).

(1) $$\begin{array}{c} I\left(x;y\right)=\iint p\left(x,y\right)\log\frac{p\left(x,y\right)}{p\left(x\right)p\left(y\right)}dxdy, \end{array}$$

where *x* and *y* are given two random variables, *p*(*x*, *y*) is the joint probability density function of *x* and *y*, *p*(*x*) and *p*(*y*) are the probability density functions of *x* and *y*, respectively. The minimum redundancy and maximum relevancy are calculated as follows, respectively.

(2) $$\begin{array}{c} \max D\left(S,c\right);D=\frac{1}{\left|S\right|}\underset{x_{i}\in S}{\sum }I\left(x_{i};c\right), \end{array}$$

(3) $$\begin{array}{c} \min R\left(S\right);R=\frac{1}{{\left|S\right|}^{2}}\underset{x_{i},x_{j}\in S}{\sum }I\left(x_{i};x_{j}\right), \end{array}$$

where *S* and |*S*| are feature subsets and the number of features contained therein, respectively, *C* is the class label, *I*(*x*_*i*_; *c*) is the mutual information between feature *i* and class label *C*, *I*(*x*_*i*_; *x*_*j*_) is the mutual information between feature *i* and feature *j*, *D* is the mean between each feature in the feature set *S* and the class label *C*, indicating the relevance between the feature set and the corresponding class label, and *R* is the size of the mutual information between the features in the feature set *S*, which represents the redundancy between the features.

The goal of the MRMR algorithm is to maximize the classification performance of the selected feature subset while minimizing the feature dimension. Therefore, it is required that the relevance between the feature subset and the label is the largest, and the redundancy between the features is the least. The minimum redundancy and maximum relevancy are constructed as follows.

(4) $$\begin{array}{c} \max\Phi_{1}\left(D,R\right),\Phi_{1}=D-R. \end{array}$$

The main process of minimum redundancy and maximum relevancy (MRMR) algorithm is as follows.

#### 2.2.1. Step 1: The First Feature Is Selected

The mutual information between all candidate variables and target variables in the clinical data of esophageal cancer patients is calculated. The feature variable with the largest mutual information is the first feature variable selected.

#### 2.2.2. Step 2: The Second Feature Is Selected

The redundancy between the selected first feature and the other features is calculated. The feature variable with the least redundancy is the second feature variable.

#### 2.2.3. Step 3: Sequential Selection of Other Features

Based on the selected two feature variables, the selection of the next feature variable is required to make the selected feature subset have the largest relevance with the target variable and the least redundancy with the selected feature. Therefore, it is necessary to satisfy the minimum redundancy and maximum relevancy criterion of Equation (4). Repeat the calculation of the criteria shown in Equation (4), and add the variables that meet the requirements to the selected feature subset in turn. When the number of selected features meets the requirements, the algorithm ends.

In order to clearly express the MRMR process, the framework of MRMR is shown in Algorithm 1.

### 2.3. Selection of Optimal Subset Combinations

The patients' 17 blood indicators, age, and TNM staging information are used as input and five-year survival status as output. The patients' indicators are reordered according to their importance by the MRMR method. The reordered dataset is put into the BP neural network [39], and the classification accuracy of the feature combination is verified by tenfold cross-validation. When the highest classification accuracy is achieved, the combination with the smallest number of features is the optimal feature combination. The result is shown in Figure 1. When the highest classification accuracy is achieved, the number of features is eleven. Therefore, the features selected in this paper are the first eleven features. The eleven features are TNM stage, BASO, Age, PT, FIB, LYMPH, RBC, TT, PLT, T stage, and GLOB.

### 2.4. Cox Regression Analysis to Verify the Correlation of Indicators

Cox regression models [40] are widely used in the medical field to analyze the effects of multiple variables on survival status and survival time. In this section, Cox regression models are used to further validate the correlation of selected features with a 5-year survival status and survival time of patients with ESCC. The SPSS 26.0 statistical software is used to make the Cox model. The survival time and survival outcome of patients with ESCC are used as dependent variables. The above eleven indicators are independent variables. The survival function at the mean of the covariate is shown in Figure 2. The results show that the *p* value of the overall score of the eleven indicators is much less than 0.05. The combination of these eleven indicators is significantly related to the survival rate of patients.

## 3. Improving the Archimedes Optimization Algorithm

### 3.1. Basic Archimedes Optimization Algorithm

The Archimedes optimization algorithm [41] (AOA) is a new metaheuristic algorithm proposed in 2020. In this algorithm, the population individuals are submerged objects, and the population position is updated by adjusting the density, volume, and acceleration of the objects. According to whether the objects collide in the liquid, AOA is divided into a global exploration stage and a local search stage. If the objects do not collide, the global exploration phase is performed. Instead, a partial development phase is performed.

#### 3.1.1. Initial Stage

In the initialization phase, AOA randomly initializes the density (*den*), volume (*vol*), and acceleration (*acc*) of individuals in the population. The current optimal individual (*x*_*best*_), optimal density (*den*_*best*_), optimal volume (*vol*_*best*_), and optimal acceleration (*acc*_*best*_) are selected. In the AOA, the individual density, volume and transfer factor TF are calculated as Equations (5)–(7), respectively.

(5) $$\begin{array}{c} den_{i}^{t+1}=den_{i}^{t}+\mathrm{rand}\times \left(den_{best}-den_{i}^{t}\right), \end{array}$$

(6) $$\begin{array}{c} vol_{i}^{t+1}=vol_{i}^{t}+\mathrm{rand}\times \left(vol_{best}-vol_{i}^{t}\right), \end{array}$$

where rand is a random number between (0,1). *den*_*i*_^*t*^ and *den*_*i*_^*t*+1^ are the densities of the individual *i* for the generation *t* and the generation *t* + 1, respectively. *vol*_*i*_^*t*^ and *vol*_*i*_^*t*+1^ are the volumes of the individual *i* in the generation *t* and the generation *t* + 1, respectively.

(7) $$\begin{array}{c} TF=\exp\left(\frac{t-t_{\max}}{t_{\max}}\right), \end{array}$$

where *t* is the current iteration number and *t*_max_ is the maximum iteration number.

When *TF* ≤ 0.5, AOA performs a global search, and the update of the individual acceleration is calculated as follows.

(8) $$\begin{array}{c} acc_{i}^{t+1}=\frac{den_{best}+vol_{best}\times acc_{best}}{den_{i}^{t+1}\times vol_{i}^{t+1}}. \end{array}$$

When *TF* = 0.5, AOA is developed locally, and the individual acceleration is updated to the following:

(9) $$\begin{array}{c} acc_{i}^{t+1}=\frac{den_{best}+vol_{best}\times acc_{best}}{den_{i}^{t+1}\times vol_{i}^{t+1}}. \end{array}$$

The acceleration of the individual is normalized to obtain Equation (10).

(10) $$\begin{array}{c} acc_{i-\mathrm{norm}}^{t+1}=u\times \frac{acc_{i}^{t+1}+\min\left(acc\right)}{\max\left(\text{acc}\right)\times \min\left(acc\right)}+l, \end{array}$$

where *acc*_*i*−norm_^*t*+1^ is the normalized acceleration of the individual *i* in the *t* generation, *u* and *l* are the parameters for adjusting the normalization range.

During the global search phase, the individual positions are updated by Equation (11).

(11) $$\begin{array}{c} x_{i}^{t+1}=x_{i}^{t}+C_{1}*\mathrm{rand}*acc_{i-\mathrm{norm}}^{t+1}*d*\left(x_{\mathrm{rand}}-x_{i}^{t}\right) \end{array}$$

where *x*_*i*_^*t*+1^ and *x*_*i*_^*t*^ are the positions of individuals in the *t* + 1 and *t* generations and *x*_rand_ is the positions of random individuals in the generation *t*. rand ∈ (0, 1) is a random number. *C*_1_ is a fixed constant. *d* is the density factor, which is calculated as follows.

(12) $$\begin{array}{c} d^{t+1}=\exp\left(\frac{t_{\max}-t}{t_{\max}}\right)-\left(\frac{t}{t_{\max}}\right). \end{array}$$

During the local development stage, the individual position is updated by Equation (13).

(13) $$\begin{array}{c} x_{i}^{t+1}=x_{\text{best}}^{t}+F\times c_{2}\times \mathrm{rand}\times acc_{i-\mathrm{norm}}^{t+1}\times d\times \left(T\times x_{\text{best}}-x_{i}^{t}\right), \end{array}$$

where *c*_2_ is a fixed constant and *F* is the direction factor that determines the update direction of the individual position, which is constructed as follows:

(14) $$\begin{array}{c} F=\left\{\begin{array}{cc} +1 & \text{if }p\leq 0.5\\ -1 & \text{if }p\;0.5, \end{array}\right. \end{array}$$

where *p* = 2 × rand − *C*_4_ and *C*_4_ is a fixed constant. *T* = *C*_3_ × *TF*, and *T* ∈ [*C*_3_ × 0.3,1.]

### 3.2. Improved Archimedean Optimization Algorithm

In the basic AOA, the update of the optimal individual of the population depends on the update of the population in each iteration. After each iteration, the optimal individual is replaced by the individual with the best fitness, and the algorithm does not actively disturb the optimal individual. When the optimal individual of the population falls into the local extremum space, the algorithm will fall into the local optimum, and the phenomenon of premature convergence will occur [42]. Therefore, this paper introduces the corresponding improvement strategy to improve the defects of the basic AOA. Firstly, Sine chaos mapping and reverse learning strategies are used to initialize the population, which can enhance the population diversity and improve the solving efficiency. Secondly, Gaussian variation and superior selection strategies are used to perturb the positions of optimal individuals, which can enhance the global search ability and help the population to jump out of the local optimum. In this paper, the improved AOA is called IAOA. The specific strategy is as follows.

#### 3.2.1. Sine Chaos Reverse Learning Initialization Strategy

The population of AOA is initialized by random generation. This leads to uneven distribution of individuals in the initial population, which affects the later iterative optimization. The Sine chaotic model [43] is a chaotic model with good randomness and ergodicity with infinite number of map foldings. Reverse learning [44] can obtain its corresponding reverse solution through the current solution. The optimal initial solution can be obtained by comparing and selecting a better solution. In this paper, the Sine chaotic strategy is used to generate an initial population with better diversity. Second, the reverse population is generated according to reverse learning. Finally, the fitness of the obtained population is calculated, and the solution with low fitness is selected as the initial population to improve the probability of obtaining the optimal initial solution. The 1-dimensional mapping expression of Sine chaos is calculated as the follows.

(15) $$\begin{array}{c} \left\{\begin{array}{c} X_{t+1}=\sin\left(2/X_{t}\right)\\ -1\leq X_{t}\leq 1, \end{array}\right. \end{array}$$

where *t* = 0, 1, 2 ⋯ , *T* and *X*_*n*_ ≠ 0.

The population *X* = {*X*_*i*_, *i* = 1, 2, ⋯.*T*}, *X*_*j*_ = {*X*_*j*_, *j* = 1, 2, ⋯dim} is obtained by mapping the Sine chaos into the solution space. The population individuals are represented as follows.

(16) $$\begin{array}{c} X_{i+1,j}=\sin\left(2/X_{i,j}\right) \end{array}$$

where *X*_*i*+1,*j*_ is the dimensional *j* value of the population *i* + 1.

The reverse population can be represented as *X*^∗^ = {*X*_*i*_^∗^, *i* = 1, 2, ⋯*T*}, *X*_*i*_^∗^ = {*X*_*ij*_^∗^, *j* = 1, 2, ⋯dim}. The reverse population individual *X*_*ij*_^∗^ can be calculated by the following.

(17) $$\begin{array}{c} X_{ij}^{*}=X_{\min j}+X_{\max j}-X_{ij}, \end{array}$$

where [*X*_min*j*_, *X*_max*j*_] is the population search dynamic boundary.

The new population {*X* ∪ *X*^∗^} is formed by the Sine chaotic population *X* and the reverse population *X*^∗^. The fitness values of the new population are ranked, and *N* individuals with the best fitness values are selected to form the initial population.

#### 3.2.2. Gaussian Operator and Superior Selection Strategy

The Gaussian operator [45, 46] is introduced in this paper in order to avoid AOA from falling into local optimum and to maintain the diversity of individuals in the population. The current optimal solution *X*_*t*_^*best*^ is subjected to Gaussian variation with certain probability *p*, and a meritocratic selection strategy is taken. The expression of the Gaussian variational operator is calculated as follows:

(18) $$\begin{array}{c} X_{i}^{t+1}=X_{i}^{t}\times \left(1+Gauss\left(\delta \right)\right), \end{array}$$

where *X*_*i*_^*t*+1^ denotes the individual position after variation and *Gauss*(*δ*) is a random variable satisfying a Gaussian distribution. The global optimal solution position is updated as follows.

(19) $$\begin{array}{c} X_{\text{best}}^{t+1}=\left\{\begin{array}{c} X_{i}^{t+1},\text{otherwise}\\ X_{i}^{t},f\left(X_{i}^{t+1}\right)>f\left(X_{i}^{t}\right)\text{ and }\mathrm{ran}{\text{d}}_{1}<p, \end{array}\right. \end{array}$$

where rand_1_ is a random variable between [0, 1], *p* is the probability of superior selection, and *f*(.) is the individual fitness value. Therefore, variational operations on the global optimal solution can avoid the algorithm from falling into a local optimum and effectively improve the search efficiency.

In order to clearly express the IAOA process, the framework of IAOA is shown in Algorithm 2.

#### 3.2.3. IAOA Validation and Comparison

In order to fully verify the effectiveness of the IAOA proposed in this paper, the improved Archimedes optimization algorithm, Archimedes optimization algorithm, sparrow search algorithm [47], and bald eagle search algorithm [48] are compared and tested under thirteen benchmark functions at the same time. The selected benchmark functions are classified into three categories. The first category is the single-peak benchmark function, as shown in F1-F5 in Table 3. The second category is the multipeak benchmark function, as shown in F6-F10 in Table 3. The third category is the multimodal benchmark function with fixed dimension, as shown in F11-F13 in Table 3. The basic parameters of the algorithm are as follows: the population size is 30, and the maximum number of iterations is 500. The other parameters within the algorithm are shown in Table 4. The experimental results are presented in Tables 5 and 6. The optimization ability of the algorithm is reflected by the optimal value and the average value, and the stability of the algorithm is reflected by the standard deviation. Firstly, for the five single-peaked functions, IAOA has higher convergence accuracy and stability compared to other algorithms. Secondly, F6 and F8 are able to reach the theoretical optimum when solving for the multipeak function. For other multipeaked functions, IAOA has the best search accuracy and stability. For fixed dimensional functions, IAOA is also better than other algorithms. Therefore, the improvement strategy proposed in this paper has improved the performance of the algorithm to some extent.

## 4. Survival Prediction Model of Patients with ESCC Based on IAOA-DBN

### 4.1. An Overview of DBN

The deep belief network (DBN) is a probabilistic generative network. It is composed by a bunch of restricted Boltzmann machines (RBMs) and a backpropagation (BP) neural network [49]. The learning process of DBN can be divided into pretraining and fine-tuning. During the pretraining process, each RBM is trained individually by an unsupervised learning algorithm in turn, and the network parameters of each layer are gradually adjusted. In the fine-tuning process, the classification labels are used as the output layer of the DBN. The BP neural network is trained sequentially from top to bottom, and the training error is propagated back to the RBM to fine-tune the parameters of all layers to reach the global optimal parameters of the DBN. The structure of DBN is shown in Figure 3.

#### 4.1.1. Pretraining of RBM

The restricted Boltzmann machine (RBM) is a neural perceptron consisting of a visible layer (*v*) and a hidden layer (*h*). Its structure is shown in Figure 4. There are bidirectional connections between the visible and hidden layers, while there is no connection between units in the same layer. In RBM, there is a weight *w* between any two connected neurons in the visible layer and the hidden layer to represent the connection strength. Each neuron has a bias coefficient *a* (for the neurons in the visible layer) and *b* (for the neurons in the hidden layer) to represent its own weight. Therefore, the energy function contained in each RBM is calculated as follows:

(20) $$\begin{array}{c} E\left(v,h;\theta \right)=-\overset{m}{\underset{i=1}{\sum }}\overset{n}{\underset{j=1}{\sum }}\omega_{ij}\nu_{i}h_{j}-\overset{m}{\underset{i=1}{\sum }}a_{i}\nu_{i}-\overset{n}{\underset{j=1}{\sum }}b_{j}h_{j}, \end{array}$$

where *θ* represents the parameter set of RBM, including the state *v*_*i*_ and bias *a*_*i*_ of the visible layer and the state *h*_*j*_ and bias *b*_*j*_ of the hidden layer, *ω*_*ij*_ is the connection weight between the visible layer node and the hidden layer node, and *n* and *m* represent the number of neurons in the visible layer and the hidden layer, respectively.

According to the energy function of the RBM, the joint distribution of the visible layer and the hidden layer is calculated as follows.

(21) $$\begin{array}{c} p\left(v,h;\theta \right)=\frac{e^{-E\left(v,h;\theta \right)}}{T\left(\theta \right)}, \end{array}$$

where *T*(*θ*) = ∑_*v*,*h*_*e*^−*E*(*v*, *h*; *θ*)^, called the normalization factor.

The independent probability distribution of the visible layer is calculated as follows.

(22) $$\begin{array}{c} p\left(v\right)=\underset{h}{\sum }p\left(v,h\right)=\frac{1}{T\left(\theta \right)}\underset{h}{\sum }e^{-E\left(v,h;\theta \right)}. \end{array}$$

There is no connection between nodes in the same layer in the RBM, so the conditional probability distribution of each neuron in the visible layer and the hidden layer is as follows:

(23) $$\begin{array}{c} p\left(h_{j}=1\left|v;\theta \right.\right)=\varepsilon \left(\overset{m}{\underset{i=1}{\sum }}\omega_{ij}v_{i}+b_{j}\right),\\ p\left(v_{i}=1\left|h;\theta \right.\right)=\varepsilon \left(\overset{n}{\underset{j=1}{\sum }}\omega_{ij}h_{j}+a_{i}\right), \end{array}$$

where *ε*(*x*) = 1/(1 + exp(*x*)) is the sigmoid function.

The goal of RBM training learning is to make the Gibbs distribution of the RBM network representation as close as possible to the distribution of the original data so that *p*(*v*) is maximized.

The network structure parameters *θ* = {*a*_*i*_, *b*_*j*_, *ω*_*ij*_} of the RBM can be obtained using the maximum likelihood estimation method, and the parameter set *θ* can be updated by the comparative scattering method, as expressed by the following.

(24) $$\begin{array}{c} L\left(\theta \right)=\overset{T}{\underset{t=1}{\sum }}\log P\left(v_{i}\left|\theta \right.\right)=\overset{T}{\underset{t=1}{\sum }}\log\underset{h}{\sum }P\left(v_{i},h\left|\theta \right.\right)=\overset{n}{\underset{i=1}{\sum }}\log f\left(v_{i}\left|\theta \right.\right)-\log T\left(\theta \right), \end{array}$$

(25) $$\begin{array}{c} \frac{\partial L\left(\theta \right)}{\partial \theta }=\overset{n}{\underset{i=1}{\sum }}\left[\frac{\partial \log f\left(v_{i}\;|\;\theta \right)}{\partial \theta }-{\langle \frac{\partial \log f\left(v\;|\;\theta \right)dv}{\partial \theta }\rangle }_{p\left(v\;|\;\theta \right)}\right], \end{array}$$

where 〈〉_*p*(*v*|*θ*)_ represents the expected value of the partial derivative under the distribution of *p*(*v* | *θ*).

The model parameter update method is as follows:

(26) $$\begin{array}{c} \omega_{ij}^{t+1}=\omega_{ij}^{t}+\frac{\alpha }{\beta }\left({\langle v_{i}h_{j}\rangle }_{\text{data}}-{\langle v_{i}h_{j}\rangle }_{\text{remodel}}\right),\\ a_{i}^{t+1}=a_{i}^{t}+\frac{\alpha }{\beta }\left({\langle v_{i}\rangle }_{\text{data}}-{\langle v_{i}\rangle }_{\text{remodel}}\right),\\ b_{j}^{t+1}=b_{j}^{\left(t\right)}+\frac{\alpha }{\beta }\left({\langle h_{j}\rangle }_{\text{data}}-{\langle h_{j}\rangle }_{\text{remodel}}\right), \end{array}$$

where 〈.〉_data_ represents the expectation of *p*(*h* | *v*) defined by the current RBM model, 〈.〉_remodel_ represents the expectation of *p*(*h* | *v*) defined by the reconstructed RBM model, *α* represents the learning rate, and *β* is the batch size.

The pretraining of DBN starts from the bottom layer. After the first RBM is trained, the current hidden layer is transformed into the visible layer of the next RBM. The network is trained layer by layer from bottom to top to avoid falling into local optimum.

#### 4.1.2. Fine-Tuning of RBM

In the fine-tuning stage, a BP neural network is constructed using the hidden layer of the last RBM and the output layer of the DBN for supervised training. The parameters of each layer are optimized from the top to the bottom to obtain the final model parameters.

### 4.2. The Proposed Parameter Optimization of DBN Based on IAOA

During the construction of DBN, the choice of hyperparameters such as learning rate *α* and batch size *β* has an important impact on the training results of DBN. However, the selection of hyperparameters in traditional DBNs mainly relies on subjective experience, which also causes the problem of insufficient training efficiency. This also leads to a decrease in the classification accuracy and model stability of DBNs. In this paper, in order to reduce the influence of human interference factors and improve the classification accuracy of DBN, the IAOA is proposed to optimize the learning rate *α* and batch size *β* of DBN. The classification error rate of DBN is used as the objective function of IAOA optimization, and the objective function is *fitnessfunction* = 1 − *classification* *error* *rate*. The larger the fitness value, the higher the classification effect of DBN. In order to clearly express the IAOA-DBN process, the framework of IAOA-DBN is shown in Figure 5.

### 4.3. Survival Prediction Model of Patients with ESCC

In this paper, eleven indicators significantly related to the survival rate of patients with ESCC are obtained through the MRMR algorithm, and these indicators are TNM stage, BASO, age, PT, FIB, LYMPH, RBC, TT, PLT, T stage, and GLOB, respectively. Eleven indicators and all indicators of the patients are used as inputs to the IAOA-DBN model, respectively, and the five-year survival rate of the patients is used as the output. A survival prediction model for esophageal cancer patients is established. The established survival prediction model for patients with ESCC is shown in Figure 6. To verify the validity of this model, the Archimedes optimization algorithm-deep belief network (AOA-DBN), sparrow search algorithm-deep belief network (SSA-DBN), particle swarm optimization-deep belief network (PSO-DBN) [50], bald eagle search-deep belief network (BES-DBN), improved Archimedean optimization algorithm-support vector machines (IAOA-SVM), and improved Archimedean optimization algorithm-backpropagation neural networks (IAOA-BPNN) are used for comparison. The initial population of AOA, SSA, PSO, and BES is uniformly set to 20, and the maximum number of iterations is 500. The dataset is divided into ten parts, and the tenfold cross-validation method is used to verify the classification accuracy of the model. The prediction results of the DBN optimized by the five optimization algorithms, IAOA-SVM, and IAOA-BPNN model are shown in Table 7.

When eleven patient indicators are used as input, the Tables 5 and 6 show that the prediction results of IAOA-DBN, AOA-DBN, SSA-DBN, PSO-DBN, BES-DBN, IAOA-SVM, and IAOA-BPNN are 89.66%, 87.46%, 88.14%, 86.78%, 87.29%, 86.27%, and 86.61%, respectively. When all patient indicators are used as input, Table 7 shows that the prediction results of IAOA-DBN, AOA-DBN, SSA-DBN, PSO-DBN, BES-DBN, IAOA-SVM, and IAOA-BPNN are 88.13%, 86.24%, 86.93%, 85.46%, 86.12%, 85.19%, and 85.32%, respectively. The comparison shows that IAOA-DBN has a high accuracy rate and can accurately predict the five-year survival rate of ESCC patients. In addition, when the input to the model is eleven indicators, the prediction results are better than using all indicators. Therefore, the MRMR-IAOA-DBN model proposed in this paper can better predict the five-year survival of patients with ESCC.

To better demonstrate the effectiveness of the proposed model, the Wisconsin Diagnostic Breast Cancer (WBCD) dataset is used for testing. In Wisconsin Diagnostic Breast Cancer (WBCD) dataset, 30 indexes of patients are used as input, and the benign and malignant tumors of patients are used as output. The dataset is divided into ten parts, and the tenfold cross-validation method is used to verify the performance of the model. The test results are shown in Table 8. From the test results, it can be seen that IAOA-DBN has higher prediction accuracy than other models. Therefore, the survival prediction model proposed in this paper can effectively predict the prognosis of cancer patients.

## 5. Conclusions

A novel survival prediction model for patients with ESCC is presented in this paper. Firstly, a minimum redundancy and maximum relevancy algorithm is used to screen out indicators significantly correlated with survival in patients, which is validated by the Cox regression analysis. Secondly, an IAOA-DBN model is proposed. The model uses IAOA to optimize the parameters in the DBN training process, which improves the stability and classification accuracy of the DBN model. Finally, the model is applied to the survival prediction model for patients with ESCC. The results of comparison with four methods verify the validity and superiority of the model. The key conclusions are expressed as follows.

1. The patients' clinical indicators are ranked by importance using the minimum redundancy and maximum relevancy algorithm, and a new subset of features is selected. The experimental results show that the new feature subset is with better prediction results than the all-feature set
2. Aiming at the problem that poor convergence accuracy and easy to fall into local optimum of AOA, an improved AOA (IAOA) is proposed in this paper. The experimental results show that the improved strategy proposed in this paper improves the performance of AOA to a certain extent
3. The learning rate *α* and batch size *β* of DBN are optimized using IAOA to obtain the optimal parameters, which improved the classification prediction accuracy and stability of the DBN model. Compared with AOA-DBN, SSA-DBN, PSO-DBN, and BES-DBN, the results verify the effectiveness and superiority of the IAOA-DBN model

## Figures and Tables

**Figure 1:** The change of classification accuracy with the number of feature variables.

**Figure 2:** Survival function at the mean of the covariate. The survival years are taken as the time, the eleven indicators obtained from minimum redundancy and maximum relevancy algorithm.

**Figure 3:** Schematic diagram of the DBN structure.

**Figure 4:** Schematic diagram of RBM structure.

**Figure 5:** The framework of IAOA-DBN.

**Figure 6:** ESCC patient survival prediction model.

**Algorithm 1:** Framework of MRMR.

**Algorithm 2:** Framework of IAOA.

**Table 1:** Population proportion information of the dataset.

Project	Category	Number of population	Percentage of population
Genders	Male	186	62.4%
	Female	112	37.6%
Ages	≤61.5	192	64.4%
	61.5	112	37.6%
T stages	T1	42	14.1%
	T2	89	29.9%
	T3	165	55.4%
	T4	2	0.6%
N stages	N0	170	57.1%
	N1	80	26.8%
	N2	34	11.4%
	N3	14	4.7%
TNM stages	1	37	12.4%
	2	139	46.6%
	3	106	35.6%
	4	16	5.4%

**Table 2:** Basic information about seventeen blood indicators.

Variable	Mean	Median (range)	Variance	Standard deviation
BASO	0.050	0 (0-1)	0.014	0.118
EO	0.144	0.1 (0-3)	0.074	0.272
FIB	379.262	362.811 (167.613-909.725)	924.038	30.398
PTL	226.289	227.5 (45-448)	62.902	7.931
ALB	42.077	42 (27-59)	25.055	5.005
HGB	137.742	139 (95-189)	227.216	15.074
WBC	6.564	6.1 (2.18-15.3)	4.077	2.019
MONO	0.406	0 (0-1)	0.091	0.301
APTT	35.929	35.1 (15.4-78.5)	62.479	7.904
GLOB	29.077	29 (17-45)	26.240	5.122
RBC	4.452	4.5 (2.93-6.04)	0.224	0.473
PT	10.322	10.2 (7-16.5)	2.834	1.684
LYMPH	1.930	1.905 (0-8)	0.479	0.692
NEUT	3.864	3.5 (0-10.6)	2.829	1.682
TP	71.070	71 (50-92)	51.971	7.209
INR	0.796	0.78 (0.45-1.64)	0.034	0.185
TT	15.569	15.7 (1.3-46.5)	6.629	2.575

The unit of WBC, LYMPH, GLOB, ALB, RBC, BASO, EO, NEUT, TP, HGB, and PLT is g/L. The unit of PT, TT, APTT is second(s). The unit of FIB is mg/L.

**Table 3:** Baseline test functions.

Funs	Name	Range	Optimum
F1	Sphere	[−100,100]^*D*^	Min = 0
F2	Schwefel2.22	[−10, 10]^*D*^	Min = 0
F3	Schwefel1.20	[−100,100]^*D*^	Min = 0
F4	Schwefel2.21	[−100,100]^*D*^	Min = 0
F5	Quartic	[−1.28,1.28]^*D*^	Min = 0
F6	Rastraign	[−32, 32]^*D*^	Min = 0
F7	Ackley	[−600,600]^*D*^	Min = 0
F8	Griewank	[−600,600]^*D*^	Min = 0
F9	Penalized 1	[−50, 50]^*D*^	Min = 0
F10	Penalized 2	[−50, 50]^*D*^	Min = 0
F11	Kowalik's	[−5, 5]^2^	3.08*E* − 04
F12	Six-hump	[−5, 5]^2^	−1.03*E* + 00
F13	Branin	[-5,10]∪[0, 15]^2^	3.98*E* − 01

**Table 4:** Algorithm parameter settings.

Algorithm	Main parameters
AOA	*C*_1_ = 2, *C*_2_ = 6, *C*_3_ = 1, *C*_4_ = 2
IAOA	*C*_1_ = 2, *C*_2_ = 6, *C*_3_ = 1, *C*_4_ = 2
SSA	ST = 0.6, PD = 0.7, SD = 0.2
BES	*a* = 10; *R* = 1.5

**Table 5:** Comparison with the results of 3 metaheuristic algorithms.

Statistics	Algorithm	F1	F2	F3	F4	F5	F6	F7
Best	IAOA	0.00**E** + 00	0.00**E** + 00	0.00**E** + 00	0.00**E** + 00	5.26**E** − 06	0.00**E** + 00	8.88**E** − 16
	AOA	4.93*E* − 126	5.61*E* − 60	1.27*E* − 100	1.55*E* − 59	9.09*E* − 05	0.00*E* + 00	8.88*E* − 16
	SSA	0.00*E* + 00	0.00*E* + 00	0.00*E* + 00	0.00*E* + 00	3.54*E* − 05	0.00*E* + 00	8.88*E* − 16
	BES	5.31*E* − 46	8.70*E* − 29	8.10*E* − 19	8.13*E* − 14	5.36*E* − 05	0.00*E* + 00	8.88*E* − 16
Mean	IAOA	0.00**E** + 00	0.00**E** + 00	0.00**E** + 00	0.00**E** + 00	9.89**E** − 05	0.00**E** + 00	8.88**E** − 16
	AOA	2.96*E* − 87	3.69*E* − 45	9.36*E* − 73	1.23*E* − 40	6.76*E* − 04	5.46*E* + 00	2.31*E* − 15
	SSA	1.58*E* − 64	3.17*E* − 29	7.63*E* − 42	1.62*E* − 45	7.50*E* − 04	0.00*E* + 00	8.88*E* − 16
	BES	4.38*E* − 41	1.17*E* − 25	4.47*E* − 04	1.51*E* − 01	2.39*E* − 03	3.64*E* + 01	8.03*E* − 03
Worst	IAOA	0.00**E** + 00	0.00**E** + 00	0.00**E** + 00	0.00**E** + 00	4.39**E** − 04	0.00**E** + 00	8.88**E** − 16
	AOA	5.17*E* − 86	1.06*E* − 43	2.74*E* − 71	2.28*E* − 39	2.35*E* − 03	1.64*E* + 02	4.44*E* − 15
	SSA	4.74*E* − 63	9.51*E* − 28	2.29*E* − 40	4.87*E* − 44	2.04*E* − 03	0.00*E* + 00	8.88*E* − 16
	BES	4.59*E* − 40	1.93*E* − 24	1.02*E* − 02	6.02*E* − 01	8.91*E* − 03	1.49*E* + 02	2.41*E* − 01
Std	IAOA	0.00**E** + 00	0.00**E** + 00	0.00**E** + 00	0.00**E** + 00	1.03**E** − 04	0.00**E** + 00	0.00**E** + 00
	AOA	8.66*E* − 64	1.94*E* − 44	5.00*E* − 72	4.44*E* − 40	5.35*E* − 04	2.99*E* + 01	1.60*E* − 15
	SSA	1.55*E* − 39	1.74*E* − 28	4.18*E* − 41	8.89*E* − 45	5.47*E* − 04	0.00*E* + 00	0.00*E* + 00
	BES	1.08*E* − 40	3.55*E* − 25	1.93*E* − 03	2.23*E* − 01	2.11*E* − 03	5.61*E* + 01	4.40*E* − 02

**Table 6:** Continuation of Table 5.

Statistics	Algorithm	F8	F9	F10	F11	F12	F13
Best	IAOA	0.00**E** + 00	1.04**E** − 13	4.32**E** − 12	3.19**E** − 04	−1.03**E** + 00	3.98**E** − 01
	AOA	0.00*E* + 00	4.85*E* − 01	2.60*E* + 00	3.35*E* − 04	−1.03*E* + 00	3.98*E* − 01
	SSA	0.00*E* + 00	5.02*E* − 06	2.21*E* − 05	3.08*E* − 04	−1.03*E* + 00	3.98*E* − 01
	BES	0.00*E* + 00	7.53*E* − 23	8.05*E* − 05	3.07*E* − 04	−1.03*E* + 00	3.98*E* − 01
Mean	IAOA	0.00**E** + 00	7.03**E** − 09	6.96**E** − 08	4.68**E** − 04	−1.03**E** + 00	3.98**E** − 01
	AOA	0.00*E* + 00	8.16*E* − 01	2.89*E* + 00	9.10*E* − 04	−1.03*E* + 00	3.98*E* − 01
	SSA	0.00*E* + 00	2.42*E* − 05	1.49*E* − 03	3.74*E* − 04	−1.03*E* + 00	3.98*E* − 01
	BES	0.00*E* + 00	1.04*E* − 02	5.03*E* − 02	3.18*E* − 03	−1.03*E* + 00	3.98*E* − 01
Worst	IAOA	0.00**E** + 00	3.86**E** − 08	3.93**E** − 07	1.32**E** − 03	−1.03**E** + 00	3.98**E** − 01
	AOA	0.00*E* + 00	1.15*E* + 00	2.99*E* + 00	5.91*E* − 03	−1.03*E* + 00	3.98*E* − 01
	SSA	0.00*E* + 00	8.30*E* − 05	1.32*E* − 02	1.22*E* − 03	−1.03*E* + 00	3.98*E* − 01
	BES	0.00*E* + 00	1.04*E* − 01	2.33*E* − 01	2.04*E* − 02	−1.03*E* + 00	3.98*E* − 01
Std	IAOA	0.00**E** + 00	1.09**E** − 08	1.16**E** − 07	1.68**E** − 04	1.79**E** − 10	5.48**E** − 07
	AOA	0.00*E* + 00	1.78*E* − 01	8.39*E* − 02	9.73*E* − 04	3.93*E* − 04	3.89*E* − 06
	SSA	0.00*E* + 00	1.87*E* − 05	3.88*E* − 03	2.53*E* − 04	4.72*E* − 08	8.16*E* − 07
	BES	0.00*E* + 00	3.16*E* − 02	7.47*E* − 02	6.86*E* − 03	1.65*E* − 08	7.18*E* − 07

**Table 7:** Comparison of different algorithms for predicting five-year survival of patients with esophageal squamous cell carcinoma.

Algorithm	10-fold cross-validation accuracy	
	Eleven indicators	All indicators
IAOA-DBN	89.66%	88.13%
AOA-DBN	87.46%	86.24%
SSA-DBN	88.14%	86.93%
PSO-DBN	86.78%	85.46%
BES-DBN	87.29%	86.12%
IAOA-SVM	86.27%	85.19%
IAOA-BPNN	86.61%	85.32%

**Table 8:** Comparison of the results of different algorithms.

Algorithm	10-fold cross-validation accuracy
IAOA-DBN	97.538%
AOA-DBN	96.974%
SSA-DBN	97.177%
PSO-DBN	96.629%
BES-DBN	96.829%
IAOA-SVM	95.602%
IAOA-BPNN	95.038%

## Data Availability

The datasets presented in this article are not readily available because the data used in the study are private and confidential data. Requests to access the datasets should be directed to Junwei Sun, junweisun@yeah.net.
